RETRACTED

# MyoD-dependent regulation of NF-κB activity couples cell-cycle withdrawal to myogenic differentiation

**DOI:** 10.1186/2044-5040-2-6

**Published:** 2012-05-19

**Authors:** Maura H Parker, Julia von Maltzahn, Nadine Bakkar, Ban Al-Joubori, Jeff Ishibashi, Denis Guttridge, Michael A Rudnicki

**Affiliations:** 1 Faculty of Health Sciences Graduate Programme, McMaster University, Hamilton, Ontario, Canada; 2 Ottawa Hospital Research Institute, Molecular Medicine Program, Ottawa, Ontario, Canada; 3 Current address: Fred Hutchinson Cancer Research Center, Clinical Research Division, Seattle, WA, USA; 4 The Ohio State University College of Medicine, Columbus, Ohio, USA; 5 Ottawa Hospital Research Institute, 501 Smyth Rd, Ottawa, ON, K1H 8L6, Canada

**Keywords:** Skeletal muscle, Myoblasts, MyoD, NF-κB, IKK, IκB, Differentiation, Myogenesis

## Abstract

**Background:**

Mice lacking MyoD exhibit delayed skeletal muscle regeneration and markedly enhanced numbers of satellite cells. Myoblasts isolated from *MyoD*^*-/-*^ myoblasts proliferate more rapidly than wild type myoblasts, display a dramatic delay in differentiation, and continue to incorporate BrdU after serum withdrawal.

**Methods:**

Primary myoblasts isolated from wild type and *MyoD*^*-/-*^ mutant mice were examined by microarray analysis and further characterized by cell and molecular experiments in cell culture.

**Results:**

We found that NF-κB, a key regulator of cell-cycle withdrawal and differentiation, aberrantly maintains nuclear localization and transcriptional activity in *MyoD*^*-/-*^ myoblasts. As a result, expression of cyclin D is maintained during serum withdrawal, inhibiting expression of muscle-specific genes and progression through the differentiation program. Sustained nuclear localization of cyclin E, and a concomitant increase in cdk2 activity maintains S-phase entry in *MyoD*^*-/-*^ myoblasts even in the absence of mitogens. Importantly, this deficit was rescued by forced expression of IκBαSR, a non-degradable mutant of IκBα, indicating that inhibition of NF-κB is sufficient to induce terminal myogenic differentiation in the absence of MyoD.

**Conclusion:**

MyoD-induced cytoplasmic relocalization of NF-κB is an essential step in linking cell-cycle withdrawal to the terminal differentiation of skeletal myoblasts. These results provide important insight into the unique functions of MyoD in regulating the switch from progenitor proliferation to terminal differentiation.

## Background

Cell survival and differentiation is regulated by NF-κB, a family of ubiquitously expressed transcription factors comprising RelA/p65, c-Rel, RelB, p50 (processed form of p105), and p52 (processed form of p100) [1]. NF-κB proteins function as homo- or heterodimers, the most common of which is the p50/p65 heterodimer. All family members contain a DNA-binding domain, a protein-protein dimerization domain, and a nuclear localization sequence (NLS). However, only RelA/p65, c-Rel, and RelB have a transactivation domain [2].

RETRACTED

Sub-cellular localization of NF-κB is regulated by ‘inhibitor of κB’ proteins: IκBα, IκBβ, and IκBϵ [3]. IκB proteins bind NF-κB, mask the nuclear localization signal, and sequester NF-κB in the cytoplasm as an inactive protein. Upon induction, IκB kinases (IKKs) phosphorylate IκB, releasing NF-κB and targeting IκB for degradation. The released NF-κB enters the nucleus, binds DNA, and regulates gene transcription. This process is normally activated by molecules such as cytokines, growth factors, and bacterial products [4].

Myogenic specification and differentiation requires the myogenic regulatory factors (MRFs), namely MyoD, Myf5, myogenin, and MRF4/Myf6 [5]. The MRFs share a highly homologous basic helix-loop-helix (bHLH) domain, which is required for DNA binding and dimerization with the E-protein family of transcription factors. MRF-E-protein heterodimers bind to the consensus E-box sequence, CANNTG, in gene promoters and regulate transcriptional activation.

In particular, MyoD and Myf5 are essential for murine skeletal muscle development [6]. However, mice lacking MyoD are viable and fertile, and display no overt phenotype [7]. This indicates that myogenic specification and differentiation during embryonic and fetal development occurs in the absence of MyoD, due to the presence of other myogenic regulatory factors, such as Myf5. Analysis of regeneration in *MyoD*^*-/-*^ muscle established an essential role for MyoD in regulating adult myogenesis. In particular, increased numbers of satellite cells and a deficient muscle regenerative process in mice lacking *MyoD* (*MyoD*^*-/-*^), or *MyoD* and dystrophin (*MyoD*^*-/-*^*:mdx*), suggests that in the absence of MyoD, satellite cells have an increased propensity for self-renewal [8].

Analysis of the differentiation kinetics of cultured *MyoD*^*-/-*^ satellite cell derived myoblasts revealed a marked delay in differentiation, characterized by reduced expression of differentiation specific markers such as myosin heavy chain, *myogeninMRF4α-actins* and *acetylcholine receptor-δ*[9-11]. Although a portion of *MyoD*^*-/-*^ cells express myosin heavy chain (MyHC), these myocytes fail to fuse and remain primarily mononuclear. Moreover, the majority of *MyoD*^*-/-*^ myoblasts display continued incorporation of bromodeoxyuridine (BrdU) into DNA after serum withdrawal, indicating DNA synthesis is maintained in the absence of mitogen stimulation.

RETRACTED

In this study, we examined the role MyoD plays in regulating cell-cycle withdrawal during terminal differentiation in adult myogenesis by undertaking a closer investigation of the molecular phenotype of *MyoD*^*-/-*^ myoblasts. We observed that *MyoD*^*-/-*^ myoblasts maintained nuclear localization of NF-κB after serum withdrawal, and displayed altered expression of NF-κB target genes. In particular, *MyoD*^*-/-*^ myoblasts failed to down-regulate *cyclin D1*, an NF-κB target gene and key mediator of cell-cycle withdrawal and differentiation in myoblasts [12,13]. Importantly, inhibition of NF-κB activity, through expression of a mutant form of IκBα (IκB-SR), rescued the differentiation of *MyoD*^*-/-*^ myoblasts. Therefore, we conclude that MyoD controls cell-cycle withdrawal by regulating the subcellular localization of the NF-κB family of transcription factors.

## Methods

### Myoblast isolation and cell culture

Myoblasts were isolated from 6 to 8 week old *wild type (WT)* Balb/C mice and *MyoD*^*-/-*^ mice and cultured as previously described [9]. To induce differentiation, the cells were washed once with PBS and transferred to differentiation medium (DMEM supplemented with 5% horse serum (Invitrogen), and 2X penicillin/streptomycin). C2C12 murine myoblasts were cultured and differentiated as previously described [14].

### Transfections and luciferase assay

C2C12 and MyoD-/- myoblasts were transfected in low serum Opti-MEM using Lipofectamine (Invitrogen, Carlsbad, CA, USA) according to the manufacturer. Reporter and expression plasmids were previously described [12], and all transfections were normalized to CMV-βGAL expression. For luciferase assays, cells were lysed in MPER (Pierce) and assays were performed as previously described [12]. MyoD siRNA was obtained from SantaCruz and transfections were performed using Lipofectamine 2000 (Invitrogen, Carlsbad, CA, USA).

### RNA isolation and RNase protection assay

RNA was isolated using TriZol Reagent (Invitrogen, Carlsbad, CA, USA) according to the manufacturer’s instructions. The RNase protection assay was performed using the RiboQuant kit according to the manufacturer’s instructions (BD Bioscience, Franklin Lakes, NJ, USA). The relative amount of radioactivity present in each band was quantitated using a Phosphorimager (GE Healthcare, Buckinghamshire, England), and the values obtained for each cyclin were normalized to the value for the GAPDH control.

### Immunoblotting and antibodies

Proteins were separated on 10% or 12% SDS-polyacrylamide gel, and transferred to a polyvinylidene fluoride membrane (Immobilon-P; Millipore, Billerica, MA, USA) according to established protocols. The antibodies used were all from Santa Cruz Biotechnology (Santa Cruz. CA, USA): anti-cyclin D1 (C-20), anti-cyclin D2 (H-289), anti-cyclin D3 (C-16), anti-cdk4 (C-22), anti-cyclin A1 (C-19), anti-cyclin E (C-19), anti-cdk2 (H-298), anti-cyclin H (C-18), anti-cdk7 (C-19), anti-NF-κB p65 (C-20), anti-Myf5 (C-19), anti-MyoD (C-20), and anti-IKKγ (FL-419). For immunoblotting, all antibodies were used according to the manufacturer’s instructions, normally at a dilution of 1:500 or 1:1,000. Goat anti-mouse and goat anti-rabbit secondary antibodies were used at 1:2,000 (BioRad, Hercules, CA, USA). Antibody-bound proteins were detected using enhanced chemiluminescence (ECL; GE Healthcare, Buckinghamshire, England) and X-OMAT 5 X-ray film.

RETRACTED

### Kinase assays

Each 10-cm plate from a differentiation time course of *WT* and *MyoD*^*-/-*^ primary myoblasts were lysed with 300 μL of NP-40 Lysis/IP buffer (50 mM Tris–HCl (pH 7.5), 150 mM NaCl, 1 mM EDTA, 2.5 mM EGTA, 1 mM DTT, 10% glycerol, 0.1 mM Na_2_VO_3_, 50 mM NaF, 20 mM β-glycerophosphate, 50 μg/mL PMSF, 2 μg/mL leupeptin, 1 μg/mL aprotinin, 10 μg/mL pepstatin). Immunoprecipitated cdk2 was incubated with 1 μg of histone H1 (Invitrogen) and 5 μCi of γ-^32^P-ATP (GE Healthcare, Buckinghamshire, England) in kinase buffer, and incubating at 30°C for 20 min. IKK kinase assays were performed as previously described using a GST-IκBα substrate [15].

### Gene expression analysis

Mouse U74Av2 GeneChip microarrays (Affymetrix, Santa Clara, CA, USA) were used to analyse gene expression in wild type and MyoD-/- primary myoblasts [16]. A list of genes related to the NF-κB pathway was defined with reference to commercial microarrays (Panomics; Superarray Bioscience, Frederick, MD, USA) and the literature. Microarray data is available from StemBase (http://www.scgp.ca:8080/StemBase/) under experiment number E223 (samples S361-4) and E59 (S78-9) and from the National Center for Biotechnology Information’s Gene Expression Omnibus (http://www.ncbi.nlm.nih.gov/geo/) under series accession number GSE3245 (GSM73053…64) and GSE3244 (GSM73026, -29, -32, -35, -38, and -41).

### Virus production and transduction

To generate ecotrophic retroviral supernatant, Phoenix-eco packaging cell lines were obtained from ATCC, cultured in DMEM with 4.5 g/L glucose (Invitrogen Life Technologies), supplemented with 100 U/mL penicillin and 100 μg/mL streptomycin, and 10% FBS (Hyclone, Logan, UT, USA), and transfected either with pBabe/Iκ (expressing IKBα-SR) or pBabe (empty vector) using lipofectamine 2000 (Invitrogen Life Technologies). Retroviral supernatant was harvested 48 h after transfection and filtered through a 0.45 μm syringe filter (Millipore). Primary proliferating *MyoD*^*-/-*^ cells were infected with diluted viral supernatant plus 8 μg/mL polybrene (hexadimetherine bromide, Sigma Aldrich, ST. Louis, MO, USA). Drug selection was conducted using 2 μg/mL Puromycin (Sigma Aldrich) for 7 days; uninfected controls were obliterated after 4 days of selection. Differentiation was induced by replacing growth medium with DMEM + 5% horse serum (Hyclone).

RETRACTED

### Animals

All animal procedures conform with the Canadian Council on Animal Care’s Guide to the Care and Use of Experimental Animals, the Animals for Research Act, and were approved by the Animal Care Committee at University of Ottawa.

## Results

### Sustained activation of NF-κB during differentiation of *MyoD*^*-/-*^ myoblasts

*MyoD*^*-/-*^ myoblasts express myosin heavy chain upon serum withdrawal, yet fail to fuse into multinucleated myotubes [9]. This phenotype is recapitulated in MyoD-expressing *IκBα-/-* fibroblasts, in which NF-κB is persistently nuclear localized [17,18]. Given that NF-κB is normally relocalized to the cytoplasm during myogenic differentiation, we sought to determine if NF-κB remains in the nucleus during induction of differentiation in myoblasts lacking MyoD. Nuclear and cytoplasmic protein extracts from a differentiation time course of *WT* and *MyoD*^*-/-*^ myoblasts were subjected to western blot analysis using an antibody specific for p65/RelA. Strikingly, *MyoD*^*-/-*^ myoblasts displayed continued nuclear localization of NF-κB (RelA/p65) after mitogen withdrawal, whereas RelA/p65 was appropriately relocated to the cytoplasm in *WT* myoblasts (Figure 1A). Furthermore we conducted immunofluorescence analyses of *WT* and *MyoD-/-* cells under growth and differentiation conditions. We observed continued nuclear localization of NF-κB (RelA/p65) in *MyoD-/-* cells during differentiation (Figure 1B) while *WT* cells displayed the expected shift in localization of NF-κB (RelA/p65) during differentiation. Furthermore, *MyoD-/-* myoblasts appear to have less cytoplasmic NF-kB than WT myoblasts in growth conditions, suggesting that NF-κB signalling is aberrant in the absence of MyoD in proliferation as well as differentiation.

**Figure 1:** **NF-κB remains localized to the nucleus after serum withdrawal in*MyoD***^***-/-***^**myoblasts.(A)** Protein was isolated from a differentiation time course of *WT* and *MyoD*^*-/-*^ primary myoblasts and a western blot using the nuclear (N) and cytoplasmic (C) fractions was performed with an antibody specific for the p65 subunit of NF-κB. A western blot with an antibody specific for α-tubulin was performed using the cytoplasmic fractions. **(B)** Immunofluorescence analysis of *WT* and *MyoD-/-* myoblasts and myotubes demonstrate that NF-κB remains localized in the nucleus in *MyoD-/-* myoblasts even after differentiation. Staining for NF-κB in red, nuclei are counterstained with DAPI (in blue). Scale bar: 20 μm.

RETRACTED

To determine if continued nuclear localization of p65 correlates with increased transcriptional activity, an NF-κB specific luciferase reporter (3xκB-Luc) was transfected into C2C12 cells lacking MyoD expression. C2C12 myoblasts transfected with *MyoD*-specific siRNA (siMyoD-C2C12) exhibited a significant decrease in MyoD expression, and resembled *MyoD*^*-/-*^ myoblasts (Figure 2A, data not shown). Luciferase activity in 3xκB-Luc-transfected siMyoD-C2C12 myoblasts was increased relative to control cells, indicating that in the absence of MyoD, RelA/p65 continued to be transcriptionally active after induction of differentiation (Figure 2B). Co-transfection with exogenous p65 enhanced activation of the 3xκB-Luc reporter, yet siMyoD cells continued to exhibit elevated NF-κB activity (Figure 2C).

**Figure 2:** **Loss of MyoD activates NF-κB.(A)** Protein isolated from C2C12 myoblasts transfected with control siRNA or siRNA specific for MyoD were analyzed by western blot using antibodies specific to MyoD and α-tubulin. **(B)** C2C12 cells transfected with control siRNA (siCont) or MyoD siRNA (siMyoD) were co-transfected with an NF-kB reporter vector (3xκB-Luc). Bars represent average luciferase activity (relative light units (RLUs)) (n = 3). Error bars represent standard deviation. **(C)** Same as B, with the addition of a p65 (NF-κB) expression vector.

To determine if expression of NF-κB target genes, or genes that participate in the NF-κB signalling pathway, were altered in the absence of MyoD, the expression profiles of *MyoD*^*-/-*^ myoblasts and *WT* myoblasts were compared using an Affymetrix microarray (Tables 1 and 2) [16]. Known NF-κB target genes were selected from genes displaying differences in expression (see http://www.bu.edu/nf-kb/gene-resources/target-genes/ for an overview). Genes that were specifically up-regulated in myoblasts lacking MyoD are tabulated in Table 1, whereas genes that were down-regulated are documented in Table 2. NF-κB target genes such as *MCP-1/CCL2/GRO-αMIP-2/CXCL1*, matrix metalloproteinases (*MMP3* and *MMP13*), *VCAM1IL-6BCL-2IL-11IGFBP-2*, and *JunB* are represented in both Tables 1 and 2, indicating that nuclear localized NF-κB was transcriptionally active in *MyoD*^*-/-*^ myoblasts. Furthermore we investigated genes involved in myogenesis. We found the following genes to be down-regulated in *MyoD*^*-/-*^ myoblasts compared to *WT* myoblasts: myogenin, Myf5, Mef2C, embryonic myosin heavy chain, MRF4/Myf6, as well as Six1.

RETRACTED

**Table 1:** **NF-κB-related genes up-regulated in*MyoD***^***-/-***^**myoblasts**

**Gene**	**RefSeq**	**Fold**	**Gene name**
Ccl2	NM_011333	166.7	Chemokine (C-C motif) ligand 2
Bgn	NM_007542	73.5	Biglycan
Mmp3	NM_010809	34.0	Matrix metallopeptidase 3
Cxcl1	NM_008176	33.0	Chemokine (C-X-C motif) ligand 1
Thbs2	NM_011581	16.9	Thrombospondin 2
Mmp13	NM_008607	9.0	Matrix metallopeptidase 13
Vcam1	NM_011693	8.2	Vascular cell adhesion molecule 1
Il6	NM_031168	8.0	Interleukin 6
Ier3	NM_133662	5.6	Immediate early response 3
Penk1	NM_001002927	4.6	Preproenkephalin 1
Pcaf	NM_020005	4.3	p300/CBP-associated factor
H2-T23	NM_010398	3.2	Histocompatibility 2, T region locus 23
Stat6	NM_009284	2.1	Signal transducer and activator of transcription 6
Ptgs2	NM_011198	2.8	Prostaglandin-endoperoxide synthase 2
Abcb1b	NM_011075	2.2	ATP-binding cassette, sub-family B (MDR/TAP), 1B
Gja1	NM_010288	2.7	Gap junction membrane channel protein alpha 1
Tnfaip3	NM_009397	2.6	Tumor necrosis factor, alpha-induced protein 3
*Bcl2*	NM_009741	2.5	B-cell leukemia/lymphoma 2

**Table 2:** **NF-κB-related genes down-regulated in*MyoD***^***-/-***^**myoblasts**

**Gene**	**RefSeq**	**Fold**	**Gene name**
Il11	NM_008350	-23.2	Interleukin 11
Igfbp2	NM_008342	-9.1	Insulin-like growth factor binding protein 2
Tlr6	NM_011604	-3.3	Toll-like receptor 6
Fos	NM_010234	-3.1	FBJ osteosarcoma oncogene
Ccnd3	NM_007632	-2.7	Cyclin D3
Cd80	NM_009855	-2.3	CD80 antigen
Junb	NM_008416	-2.3	Jun-B oncogene
*Selp*	NM_011347	-1.9	Selectin, platelet

### *MyoD*^*-/-*^ myoblasts maintain expression of cyclin D1 and D2 after serum withdrawal

*MyoD*-null myoblasts continue to proliferate in the absence of mitogens, indicating that cell-cycle modulators, such as cyclins, may be aberrantly expressed and/or regulated. Given that RelA/p65 specifically regulates expression of *cyclin D1* in myoblasts we hypothesized that persistent activation of RelA/p65 would result in continued expression of *cyclin D1* in *MyoD*^*-/-*^ myoblasts, even after serum withdrawal [12].

In order to investigate changes in important cell-cycle genes in the absence of MyoD, RNA was isolated from a differentiation time course of *MyoD*^*-/-*^ and *WT* primary myoblasts, and the relative expression level of a variety of cyclins was determined using an RNase protection assay. The relative amount of mRNA present for each cyclin was quantitated using a phosphorimager, and normalized to a *GAPDH* control. Figure 3A and 3C show resulting autoradiographs of polyacrylamide gels, and Figure 3B and 3D graphically depicts quantitation of the results. *MyoD*^*-/-*^ myoblasts exhibited a higher level of *cyclin D1* and *D2* mRNA, and a lower level of *cyclin D3* and *cyclin G1* mRNA when compared to WT myoblasts (Figure 3A, 3B, and 3F). However, neither *cyclin E* nor *cyclin H* mRNA was affected by the absence of MyoD (Figure 3C and 3D).

RETRACTED

**Figure 3:** ***MyoD***^***-/-***^**myoblasts maintain cyclin D expression after serum withdrawal.(A, C)** RNA was isolated from a differentiation time course of *WT* and *MyoD*^*-/-*^ primary myoblasts and an RNase protection assay was performed with the indicated probes. The protected ^32^P-labeled fragments were separated on a polyacrylamide gel, the gel dried and exposed to X-ray film. **(B, D)** The amount of each protected fragment was quantitated using a phosphorimager. The values obtained were normalized relative to the GAPDH control and the L32 control, and graphed as a function of the number of days in differentiation medium (DM), n = 3. **(E)** Nuclear protein was isolated from a differentiation time course of *WT* and *MyoD*^*-/-*^ primary myoblasts and a western blot was performed with the indicated antibodies. **(F)** Quantitative real-time PCR for Cyclin D3 of *WT* and *MyoD-/-* myoblasts, n = 3.

To determine if changes in mRNA expression are translated into changes in protein levels, nuclear protein extracts were isolated from a similar differentiation time course and analyzed by western blot analysis. In accord with RNase protection assay results, *MyoD*^*-/-*^ myoblasts displayed a higher level of cyclin D1 and D2 protein in the nucleus, and continued expression of both cyclins after mitogen withdrawal (Figure 3E). Expression of cyclin D3 protein, on the other hand, was not altered in the absence of MyoD. Taken together, these data imply that persistent activation of RelA/p65 is responsible for expression of cyclin D1 in *MyoD*^*-/-*^ myoblasts after serum withdrawal.

pRb is also phosphorylated by cyclin E-cdk2, and this phosphorylation is required for S-phase entry [19]. Moreover, forced expression of cyclin E bypasses the need for cyclin D/cdk4 activity in cell-cycle progression from G1 to S phase [20,21]. Expression of *cyclin E* mRNA was not altered in the absence of MyoD, indicating that the increase in cyclin D1 expression is not inducing cell-cycle progression through stimulation of E2F activity on the *cyclin E* promoter (Figure 3C and D).

However, overexpression of cyclin D1 may also inhibit MRF activity and myogenic differentiation through a mechanism independent of pRb or MyoD phosphorylation [22-24]. Indeed, a hypophosphorylated mutant of pRb (pRbΔp35; EF), which induces cell-cycle withdrawal, is unable to rescue cyclin D-dependent inhibition of muscle-specific gene expression (MH Parker, MA Rudnicki, unpublished observations).

RETRACTED

### Loss of MyoD stimulates S-phase entry

Although expression of *cyclin E* mRNA was not altered (Figure 3C and 3D), western blot analysis of protein extracts from a differentiation time course of wild type and *MyoD*^*-/*^-myoblasts displayed an increased level of cyclin E protein in the nucleus (Figure 4A). This may be the result of increased stability of cyclin E protein, or of prolonged nuclear localization after mitogen withdrawal. The level of nuclear cdk2 protein was also elevated, and more importantly, appeared to be the slower migrating, activated form. In order to determine if cdk2 activity was maintained after mitogen withdrawal, a kinase assay was employed using protein extracts from the same differentiation time course of wild type and *MyoD*^*-/-*^ myoblasts. As expected, elevated levels of cdk2 correlated with increased cdk2 kinase activity (Figure 4B).

**Figure 4:** ***MyoD***^***-/-***^**myoblasts enter S-phase more readily than WT myoblasts.(A)** Western blot was performed using the indicated antibodies and nuclear protein isolated from a differentiation time course of *WT* and *MyoD*^*-/-*^ primary myoblasts. **(B)** Cdk2 was immunoprecipitated from protein extracts of a differentiation time course of *WT* and *MyoD*^*-/-*^ primary myoblasts, and assayed for kinase activity using histone H1 and γ-^32^P-ATP as substrate. **(C)** Proliferating *WT* and *MyoD*^*-/-*^ myoblasts were fixed in ethanol and DNA stained with propidium iodide (PI). Cells were analyzed for DNA content by FACS analysis. The percentage of cells in each phase of the cell cycle is indicated.

To determine if increased cdk2 kinase activity forced cells to enter S-phase more readily, proliferating *MyoD*^*-/-*^ and *WT* myoblasts were fixed and analyzed for DNA content using fluorescence activated cell sorting (FACS). As expected, *MyoD*^*-/-*^ myoblasts displayed a two-fold increase in the number of cells in S-phase (23% of *MyoD*^*-/-*^ myoblasts compared to 12% of *WT* myoblasts; Figure 4C). This increase in the proportion of *MyoD*^*-/-*^ myoblasts in S-phase was accompanied by a decrease in the proportion of cells in the G1 phase of the cell cycle (68% of *MyoD*^*-/-*^ cells compared to 84% of *WT* cells). Therefore, in the absence of MyoD, myoblasts enter into S-phase more readily, likely as a result of increased cyclin E-cdk2 activity.

### Inhibition of NF-κB restores differentiation of *MyoD*^*-/-*^ myoblasts

Skeletal muscle differentiation requires both cell-cycle withdrawal and muscle-specific gene expression. *MyoD*^*-/-*^ myoblasts fail to withdraw from the cell cycle, as evidenced by continued DNA synthesis after induction of differentiation [9]. Given that *MyoD*-null myoblasts aberrantly maintain transcriptionally active RelA/p65 after serum withdrawal, we hypothesize that persistent activation of RelA/p65 is responsible for the failure to exit the cell cycle. Moreover, we propose that the inability to induce cell-cycle withdrawal is directly responsible for the delay in differentiation in *MyoD*^*-/-*^ myoblasts.

RETRACTED

IκB kinases (IKKs) phosphorylate IκB, resulting in degradation of IκB and nuclear localization of RelA/p65 [3]. To determine if IKK activity is aberrantly maintained in *MyoD*-null myoblasts after induction of differentiation, IKK was immunoprecipitated from *MyoD*^*-/-*^ and wild type myoblast protein extracts and kinase activity assayed using GST-IκBα and γ-^32^P-ATP as substrate. *MyoD*-null myoblasts displayed approximately 2-fold greater IKK activity, as compared to WT myoblasts (Figure 5A).

**Figure 5:** **Elevated IKK activity in*MyoD***^***-/-***^**myoblasts is responsible for increased NF-κB activity.(A)** Kinase assay (KA): IKK was immunoprecipitated from protein extracts of *WT* (MyoD^+/+^) and *MyoD*^*-/-*^ primary myoblasts, and assayed for kinase activity using GST-IκBα and γ-^32^P-ATP as substrate. Immunoblot (IB): IKK was immunoprecipitated from protein extracts of *WT* (MyoD^+/+^) and *MyoD*^*-/-*^ primary myoblasts, and assayed by western blot using an antibody specific for IKKγ. **(B)***MyoD*^*-/-*^ myoblasts were transfected with vector control, vector expressing a dominant negative mutant IKKβ (IKKβ DN) or a non-phosphorylatable mutant of IkBα (IκB-SR), in addition to an NF-κB reporter (3xκB-Luc). Bars represent average luciferase activity (relative light units (RLUs)) (n = 3). Error bars represent standard deviation.

If increased IKK activity results in RelA/p65 activation, then inhibiting IKK should inhibit NF-κB transcriptional activity. Treating *MyoD*^*-/-*^ myoblasts with a chemical inhibitor of IKK (data not shown), or expressing a dominant negative mutant of IKKβ (IKKβ DN), resulted in decreased activity of 3xκB-Luc, indicating that elevated IKK activity is in part responsible for persistent NF-κB transcriptional activity (Figure 5A). Therefore, to target RelA/p65 directly, a non-phosphorylatable mutant form of IκBα (IκBα-SR) was expressed, which is resistant to targeted degradation and prevents nuclear localization of NF-κB. Indeed, expression of IkBα-SR in *MyoD*^*-/-*^ myoblasts inhibited 3xκB-Luc activity, indicating that NF-κB was directly repressed (Figure 5B). Moreover, expression of IκBα-SR in *MyoD*^*-/-*^ myoblasts down-regulated expression of cyclin D1 and cdk2 upon initiation of differentiation (Figure 6C). This strongly suggests that sustained nuclear localization of RelA/p65 in the *MyoD*-null myoblasts is responsible for cellular proliferation after serum withdrawal.

RETRACTED

**Figure 6:** **Nuclear localization of NF-κB inhibits terminal differentiation.(A)***MyoD*^-/-^ myoblasts were infected with empty capsid (pBABE) or virus expressing IκBα-SR (pBABE-IkB). Protein extracts from proliferating infected cells and uninfected cells (control) were analyzed by western blot analysis using an antibody specific to IκBα. **(B)***MyoD*^*-/-*^ myoblasts were infected with empty capsid (pBABE) or virus expressing IκBα-SR (pBABE-IkB). Proliferating cells (GM), or cells induced to differentiate for 5 days, were fixed and assessed for myosin heavy chain (MyHC) expression (in green). Nuclei were visualized using DAPI (in blue). **(C)** Fusion index of myotubes from *MyoD*^*-/-*^ cells either infected with a control (pBABE) or an IκBα-SR (pBABE-IkB) expressing virus, n = 5, ** = *P* < 0.01, *** = *P* < 0.001. **(D)***MyoD*^*-/-*^ myoblasts were infected with empty capsid (pBABE) or virus expressing IκBα-SR (pBABE-IkB). Protein extracts from a differentiation time course of infected and uninfected cells were analyzed by western blot analysis using the antibodies indicated

Importantly, inhibition of NF-κB activity also induced expression of myogenin and myosin heavy chain one day after serum withdrawal, and resulted in the formation of multinucleated myotubes (Figure 6B to 6D). This is in contrast to *MyoD*^*-/-*^ myoblasts infected with control virus, which up-regulated myogenin and myosin heavy chain to a much lower extent, even 5 days after serum withdrawal (Figure 6D, DM5). Additionally we examined the fusion index of myotubes of control and IκBα-SR expressing *MyoD-/-* cells at days 3 and 5 after serum withdrawal. Overexpression of IκBα-SR led to a significantly increased fusion index as well as to more differentiation in general (Figure 6B and 6C).

It is interesting to note that IκBαSR-expressing *MyoD*^*-/-*^ cells up-regulate expression of Myf5 during proliferation and early differentiation (Figure 6D). Increased expression of Myf5 may compensate for the lack of MyoD, and may be responsible for the induction of differentiation specific genes, such as myogenin and myosin heavy chain, after cell-cycle withdrawal. This is consistent with the fact that embryonic and fetal skeletal muscle development is able to occur in *MyoD*^*-/-*^ mice [7].

## Discussion

Finding the specific MyoD-regulated gene product that links cell-cycle withdrawal and terminal myogenic differentiation has been hitherto elusive. In this study, we demonstrate that continued proliferation and inhibition of differentiation in *MyoD*-null myoblasts is due to persistent nuclear localization of RelA/p65. Expression of a non-phosphorylatable mutant of IκBα (IκBα-SR), which induces cytoplasmic retention of RelA/p65, down-regulated expression of cyclin D1 in *MyoD*^*-/-*^ myoblasts, and resulted in the formation of multinucleated myotubes. Therefore, inhibition of RelA/p65 activation was able to substitute for MyoD expression during myogenic differentiation. Taken together, this indicates that RelA/p65 provides the link between MyoD-induced cell-cycle withdrawal and differentiation.

RETRACTED

MyoD is postulated to initiate expression of p21 and p57, inhibitors of cdk2 and cdk1 kinase activity [25-27]. Moreover, mice lacking *p21* and *p57* are phenotypically similar to *myogenin* knockout mice, in that they lack differentiated myofibers [28]. These data suggest that myogenic cell-cycle withdrawal and differentiation requires MyoD-dependent induction of cdk inhibitor expression. However, *MyoD*^*-/-*^ myoblasts have a similar level of *p21* mRNA as compared to *WT* myoblasts, and mice lacking *p21* display no apparent muscle abnormalities [9,29]. Therefore, we propose that adult satellite cells utilize an alternate or additional mechanism for inducing cell-cycle withdrawal during terminal differentiation: down-regulation of RelA/p65 activity.

Notably, *MIP-2/CXCL1/GRO-α* and *IL-6*, which were upregulated 33-fold and 8-fold, respectively, in *MyoD*^*-/-*^ myoblasts, are associated with constitutive activation of NF-κB, and promote tumor growth and progression [30]. Importantly, *IGFBP-2*, which binds IGFs and specifically inhibits IGF-dependent myogenic cell proliferation, was down-regulated 9.1-fold in *MyoD*^*-/-*^ myoblasts [31-35]. Therefore, in the absence of MyoD, myoblasts are programmed to proliferate as a result of maintaining growth factor signaling. This is consistent with data demonstrating that *MyoD*^*-/-*^ myoblasts have an increased propensity for proliferation and self-renewal.

*Biglycan* and *thrombospondin 2*, two genes that were up-regulated in *MyoD*^*-/-*^ myoblasts (73.5-fold and 16.9-fold, respectively), are extracellular matrix components that play important roles in scaffolding and signal transduction during myogenic regeneration. In particular, biglycan binds TGF-β, and plays an important role in mediating TGF-β signaling in responding cells [36,37]. This is important given that TGF-β inhibits myogenic differentiation and induces expression of *cyclin D1*[22]. Taken together, these data strongly suggest that NF-κB regulates expression of genes important for inducing cell proliferation.

RETRACTED

During normal differentiation of myoblasts, NF-κB is relocalized to the cytoplasm and DNA-binding activity decreases within 24 h of serum withdrawal [12,18]. Differentiation is accelerated in myoblasts expressing a non-phosphorylatable form of IκBα (IκBαSR), which is unable to be degraded, thus inhibiting NF-κB (p65) nuclear localization [12]. Furthermore, these IκBαSR-expressing myoblasts proliferate less rapidly and down-regulate expression of *cyclin D1*. In contrast, *IκBα*^*-/-*^ mouse embryonic fibroblasts (MEFs) infected with a MyoD-expressing retrovirus maintain NF-κB nuclear localization, resulting in the formation of fewer myotubes that are smaller and incorporate fewer nuclei [17]. Our experiments explain mechanistically why *MyoD*-null myoblasts display a phenotype similar to that of MyoD-infected *IκBα*^*-/-*^ MEFs.

During myogenic regeneration, satellite cells are activated and proliferate prior to initiating differentiation. Increased numbers of satellite cells and a deficient muscle regenerative process in *MyoD*^*-/-*^ mice suggest that in the absence of MyoD, satellite cells have an increased propensity for self-renewal rather than differentiation [38]. In light of the data presented here, we conclude that RelA/p65 plays an important role during the myoblast to myotube transition during adult myogenesis. Indeed, treatment of *mdx* mice with a cell permeable peptide inhibitor of IKK, which specifically inhibits NF-κB activity, restores regeneration, as evidenced by a greater number of newly formed myofibers, and increased muscle tetanic force [39].

Failure to induce myogenic differentiation is also illustrated in rhabdomyosarcoma (RDS), one the most common childhood solid tumors. RDS is characterized by inhibition of MyoD activity and concomitant failure to withdraw from the cell cycle and differentiate. This study suggests that loss of MyoD activity in RDS cells may cause aberrant nuclear localization of NF-κB, resulting in sustained cyclin D1 expression. As such, inhibiting IKK and stabilizing IκBα may play a valuable role in inhibiting proliferation and inducing differentiation in RDS cells.

During myogenesis, cytoplasmic re-localization of RelA/p65 after mitogen withdrawal plays a key role for down-regulating *cyclin D* expression, inducing cell-cycle withdrawal and activating differentiation-specific gene expression. Therefore, the regulation of NF-κB is essential in the induction of myogenic differentiation. Our experiments define the mechanistic link between MyoD and NF-κB that acts to couple cell-cycle withdrawal to terminal differentiation.

## Conclusion

We have demonstrated that NF-κB, a key regulator of cell-cycle withdrawal and differentiation, aberrantly maintains nuclear localization and transcriptional activity in *MyoD*^*-/-*^ myoblasts. Cyclin D is consequently maintained during serum withdrawal, inhibiting progression through myogenic differentiation. Sustained nuclear localization of cyclin E, and a concomitant increase in cdk2 activity maintains S-phase entry in *MyoD*^*-/-*^ myoblasts even in the absence of mitogens. Forced expression of IκBαSR, a non-degradable mutant of IκBα, rescued the deficit indicating that inhibition of NF-κB is sufficient to induce terminal myogenic differentiation. Therefore, MyoD-induced cytoplasmic relocalization of NF-κB is an essential step in linking cell-cycle withdrawal to terminal differentiation.

RETRACTED

## Abbreviations

bHLH, Basic helix-loop-helix; BrdU, Bromodeoxyuridine; FACS, Fluorescence activated cell sorting; IKK, IκB kinase; MEF, Mouse embryonic fibroblast; MRF, Myogenic regulatory factors; MyHC, Myosin heavy chain; NLS, Nuclear localization sequence; WT, Wild type; siRNA, Small interfering RNA.

## Competing interests

The authors declare no competing interests.

## Authors’ contributions

MHP and NB carried out the experiments and drafted the manuscript. BAJ and JM carried out the rescue experiments. JI performed the microarray experiment. DG provided essential reagents and participated in the design and coordination of the study. MAR conceived of the study, and participated in its design and coordination and helped to draft the manuscript. All authors read and approved the final manuscript.
